# The role of *CRP* and *ATG9B* expression in clear cell renal cell carcinoma

This article has been retracted.

**DOI:** 10.1042/BSR20171082

**Published:** 2017-11-15

**Authors:** Zheng Ma, Zengguang Qi, Zhengfei Shan, Jiangsong Li, Jing Yang, Zhonghua Xu

**Affiliations:** 1 Department of Urology, the Affiliated Yantai Yuhuangding Hospital of Qingdao University, Yantai 264000, Shandong, China; 2 Department of Organ Transplantation, the affiliated Yantai Yuhuangding Hospital of Qingdao University, Yantai 264000, Shandong, China; 3 Department of Urology, Liaocheng People’s Hospital, Liaocheng 252000, Shandong, China; 4 Department of Urology, Guanxian Center Hospital, Liaocheng 252500, Shandong, China; 5 Department of Pediatrics, Liaocheng People’s Hospital, Liaocheng 252000, Shandong, China; 6 Department of Urology, Qilu Hospital of Shandong University, Jinan 250012, Shandong, China

**Keywords:** ATG9B, clear cell renal cell carcinoma (CCRCC), CRP, cell apoptosis

## Abstract

The purpose of the study is to investigate the correlation between the expression of C-reactive protein (*CRP*) and autophagy-related 9B (*ATG9B*) and pathological features of clear cell renal cell carcinoma (CCRCC) patients. We also intended to explore the effects of manipulated expression of *CRP* and *ATG9B* on the apoptosis and cell cycle progression of CCRCC cell line. *ATG9B* expression in CCRCC tissues and adjacent renal tissues was analyzed by immunohistochemistry (IHC). Gene expression was determined at transcription and translational levels using real-time quantitative PCR (RT-qPCR) and Western blot. The association between *CRP/ATG9B* expression and clinical-pathological parameters including age, gender, pathological grades, TNM stage and distant metastasis of the patients was assessed by correlation analysis. siRNA and overexpression plasmids construction were used to manipulate the expression of *CRP* in human CCRCC cell line 786-O. Cell apoptosis and cell cycle progression were determined using flow cytometry (FCM) and Hoechst 33258 staining. *CRP* expression correlates with *ATG9B* expression. The expression of *CRP* and *ATG9B* are significantly correlated with TNM staging, distant metastasis, and survival time of CCRCC patients. A high-level of *CRP* indicates a poor overall survival (OS). In addition, *CRP* expression influences cell cycle and apoptosis of CCRCC cells. The study reveals that *CRP* might be a CCRCC development promoter. In addition, there is a close relationship between *CRP* and *ATG9B* in CCRCC carcinogenesis.

## Introduction

Renal cell carcinoma (RCC) is the most common substantial lesion within kidney [1], constituting 2–3% of adult malignancies [2] and 85% of primary renal tumors [3]. It commonly spreads to lungs, liver, bones, brain, adrenals, and lymph nodes, but seldom to skin, thyroid, and pancreas [4]. Clear cell renal cell carcinoma (CCRCC), as a subtype of RCC, accounts for ~75% of RCC [5]. Forty percent of CCRCC patients would eventually die of carcinoma development [6]. CCRCC shows the highest fatality rate amongst the common urologic malignancies [7]. Over 10000 patients die from kidney cancer each year, however, systemic treatment of RCC has improved vastly in the last two decades [8]. The pathogenesis of the most common type of RCC, CCRCC has been better understood. Therapies with high rates of response, longer progression-free survival such as anti-angiogenic drugs targetting vascular endothelial growth factor (VEGF) and its receptors, and mechanistic target of rapamycin (mTOR) inhibitors have been used [9].

The C-reactive protein (*CRP*) is located on chromosome 1q23.2 and encodes protein that belongs to the pentaxin family. *CRP* is a plasma protein mainly generated in liver and activated by interleukin 6 (IL-6) [10]. It is a prognostic factor for survival and recurrence of different types of cancers including mammary, prostatic, colonic, hepatocellular, bone, and upper aerodigestive tract (UADT) tumors [11–14]. Additionally, a previous meta-analysis has shown that high serum level of *CRP* (>1.0 mg/dl) is correlated with increased hazard of lung cancer and possibly breast, prostate, and colorectal cancers [15]. Furthermore, recent studies have revealed that *CRP* expression is significantly associated with overall survival (OS) time of patients with RCC [16–19]. However, whether abnormal *CRP* expression is associated with CCRCC pathogenesis, metastasis, and OS remains to be clarified.

The autophagy-related 9B (*ATG9B*), located on chromosome 7q36.1, belongs to the *ATG* family. A previous study has shown that *ATG9B* expression is tissue specific, that is *ATG9B* is abundant in organs such as placenta and ovary but minimum in lung, testis, liver, muscle, brain, and pancreas [20]. The methylation of *ATG9B* promoter may interrupt the autophagy signal pathway and influence the invasive ductal carcinoma (IDC) development [21]. Similarly, Kang et al. [22] discovered that the mutation of *ATG9B* is common in human gastric and colorectal cancers and it can be closely related to stomach and colorectal carcinogenesis, suggesting that *ATG9B* mutation may promote neoplasm development by deregulating autophagy. Whats more, *ATG9B* interacted with p38IP and regulated by p38α mitogen-activated protein kinase (MAPK) pathway, which then influenced the trafficking of *ATG9B* and therefore the autophagy process in a mammalian system [23,24]. Autophagy is closely related to cancer development including CCRCC [25,26]. However, the relationship between *ATG9B* expression and CCRCC pathogenesis, metastasis, and OS remains to be clarified as well.

Previous studies have shown us the aberrant expression of *CRP* and *ATG9B* and their relationship with various human diseases especially cancer development including CCRCC. Yet, the influence of their expression on CCRCC progression remains further elaborated. Our study here aimed to explore the relationship between *CRP* and *ATG9B* expression with CCRCC pathogenesis, metastasis, and survival as well as the role they play in CCRCC using *in vitro* experiments.

## Materials and methods

### Tissue specimens

One hundred and eighty five CCRCC tissues and normal adjacent tissues were collected from CCRCC patients in the Urology Center of Liaocheng People’s Hospital between 2013 and 2016. All tissues were frozen in liquid nitrogen immediately and were stored at −80°C. No patients had received any adjuvant treatments, such as radiotherapy or chemotherapy before surgery. Written informed consents were obtained from all the participants. The study had been approved by the Ethics Committee of Liaocheng People’s Hospital.

### Cell culture and siRNA transfection

CCRCC cell line (786-O) was purchased from American Type Culture Collection (ATCC; Manassas, VA, U.S.A.). All cells were placed in Dulbecco’s modified Eagle’s medium (DMEM; Gibco, Life Technologies, Darmstadt, Germany) which contains 10% FBS (HyClone, Logan, UT), penicillin (100 U/ml), and streptomycin (100 mg/ml). All were stored at 37°C in a humidified atmosphere containing 5% CO_2_. SiRNA-1 and siRNA-2 were synthesized by Suzhou GenePharma Co., Ltd. (Suzhou, China). Twenty-four hours before transfection, the 786-O cells were seeded in the DMEM medium with 10% FBS without antibiotics so the cells grew to 90% confluence. siRNA–Lipofectamine 2000 complexes were prepared. Briefly, siRNA-1 and siRNA-2 were resuspended in 1× siRNA buffer to reach a final concentration of 1 μM. One microliter of siRNA solution was added to 100 μl of serum-free medium to mix. Lipofectamine 2000 reagent (0.5 μl) was added to 25 μl serum-free medium. siRNA medium and diluted Lipofectamine 2000 reagent were incubated together for 20 min at room temperature to allow complex formation. The old medium was removed after 4–6 h. The complexes were added to each well. Cells were then harvested 24 h after transfection. The siRNA sequences were provided in Supplementary Table S1. SiRNA-1 and siRNA-2 were both used to knockdown *CRP*, yet they had different sequences.

### ELISA

CRP human ELISA Kit (ab99995, Abcam, Boston, MA, U.S.A.) was purchased for conducting ELISA. All materials were prepared at room temperature prior to use. One hundred microliters of standards and tissue samples were added to wells. The wells were covered and incubated for 2.5 h. The solution was discarded and the wells were washed three times by adding 300 μl 1× wash solution into each well. Any remaining liquid was removed completely. One hundred microliters of 1× biotinylated anti-human CRP detector antibody was added to each well. The antibody was incubated for 1 h. Then the solution was discarded and the wells were washed three times by adding 300 μl of 1× wash solution into each well. One hundred microliters of 1× HRP-streptavidin solution to each well and incubated for 45 min. The solution was removed completely. One hundred microliters of TMB One-Step substrate reagent was added to each well and incubated for 30 min in the dark. Last, 50 μl of stop solution was added to each well. The optimal density was read at 450 nm immediately.

### RNA extraction and real-time quantitative PCR

Total mRNAs of stored human CCRCC tissues and cells were extracted using TRIzol reagent (Invitrogen, Carlsbad, CA, U.S.A.) following the manufacturer’s instructions. Reverse-transcribed cDNA synthesis was performed with PrimeScript RT Reagent Kit (TaKaRa, Dalian, China). Real-time quantitative PCR (RT-qPCR) was conducted using miSYBR-Green PCR kit (TransGen Biotech, China) according to manufacturer’s protocols. Data were evaluated using SDS 2.2 software. GAPDH acted as the internal control. The expressions of *CRP* and *ATG9B* were quantitated using 2^−ΔΔ*C*^_t_ method. The primer sequences are listed in Table 1.

**Table 1:** RT-qPCR primer sequences

Gene name	Primers (5′–3′)
*CRP*	F: TGTGAGCCAGAAAAACAAGCAAA
	R: GGTATGGGGGTGGGGTCTAA
*ATG9B*	F: TGTGAGCCAGAAAAACAAGCAAA
	R: GGTATGGGGGTGGGGTCTAA
*GAPDH*	F: TGTGAGCCAGAAAAACAAGCAAA
	R: GGTATGGGGGTGGGGTCTAA

### Immunohistochemical staining

Three micrometers thick paraffin-embedded histotomy was soaked in xylene to dewax twice for 20 min, hydrated in gradient ethanol (100, 90, 80, and 70%) for 7 min. The specimens were then rinsed in the tap water three times, 3 min each time. The tissue sections were boiled with sodium citrate buffer for 5 min. The sections were then cultured in 3% H_2_O_2_ for 10 min to prevent endogenous peroxidase activities. The slices were then rinsed using PBS three times (5 min each time) and sealed in 10% serum for 10 min at room temperature to avoid non-specific binding. The tissue sections were subsequently incubated with primary antibodies anti-*CRP* antibody (ab31156, 5 µg/ml, Abcam, Boston, MA, U.S.A.) and anti-*ATG9B* antibody (ab117591, 5 µg/ml, Abcam, Boston, MA, U.S.A.). After incubation at 4°C overnight with Galectin-3, the serum was discarded and the sections were mixed with biotinylated secondary antibodies for 10 min after being washed in PBS three times (5 min each time). Afterwards, the tissue sections were cultured with streptavidin-horseradish peroxidase (SA-HRP) for another 10 min and rinsed with PBS for 5 min, three times. Finally, after diluting with 3,3′-diaminobenzidine (DAB), the sections were blended with Mayer’s Hematoxylin (Merck, Darmstadt, Germany), gradient ethanol (95, 85, and 75%) for 3 min, respectively as well as absolute ethanol for 10 min and dehydrated in xylene twice, each time 5 min. The criteria immunohistochemical (IHC) staining records showed were: no expression (0 represents without staining), low expression (1 represents more than 30% of cells weakly stained), or high expression (2 represents more than 30% of cells strongly stained).

### Western blot

Cells were washed with PBS, scraped from the dishes and centrifuged at 12000 r.p.m. at 4°C for 15 min. Cell lysates were prepared with radioimmunoprecipitation assay (RIPA) buffer. The supernatants were collected and protein concentration was determined using the BCA assay (Beyotime, Shanghai, China). Proteins were separated by SDS/PAGE (Bio–Rad, Hercules, CA, U.S.A.), transferred on to PVDF membranes (Invitrogen, Gaithersburg, MD, U.S.A) for Western blot analysis following the manufacturer’s guidelines. PVDF membranes were sealed using 5% skim milk for 1 h at room temperature, and then incubated with primary antibodies anti-CRP (ab31156, 5 µg/ml, Abcam, Boston, MA, U.S.A.) and anti-ATG9B (ab117591, 2 µg/ml, Abcam, Boston, MA, U.S.A.). After culturing with primary antibodies overnight at 4°C, secondary antibodies (1:1000) were added for another 1-h incubation at room temperature. The membranes were washed three times with TBS-Tween (TBST). The immunoreactive protein bands were visualized using G: Box XR5 and the membranes were subsequently exposed.

### Hoechst 33258 staining

786-O cells were seeded on cover slips in 24-well plates. After transfection for 48 h, cells were mixed with 4% paraformaldehyde at room temperature for 5 min. The cells were then permeabilized using 0.2% Triton X-100 solution with PBS for another 5 min, and rinsed with PBS. Then, 5% BSA was used to block the cells at room temperature for 2 h, after which they were rinsed with PBS three times (5 min each time). The cells were then stained with 0.5 ml Hoechst 33258 in dark for 5 min and rinsed in PBS. Finally, they were coverslipped with aqueous mounting medium (Dako Faramount, Shanghai, China) for later observation.

### Apoptosis assay

Flow cytometry (FCM) was employed to analyze the apoptosis in CCRCC cells. Cells were collected in logarithmic growth phase, placed in a 96-well plate and preincubated for 24 h in a CO_2_ incubator. Single-cell suspensions were fixed with 70% alcohol and then rinsed twice with PBS and binding buffer was employed to resuspend cells. For Annexin V staining, 5 μl Annexin V-PE, 5 μl 7-AAD staining and binding buffer of 10 mM HEPES/NaOH (pH 7.4), 140 mM NaCl, and 2.5 mM CaCl_2_ were added to samples, which were incubated for 15 min at room temperature in dark and analyzed by a flow cytometer (FACSCanto II, BD Biosciences). The data were analyzed using FlowJo software (LLC, Ashland, OR, U.S.A.). Three experiments were performed in triplicate. Apoptotic cells that were positive of Annexin V-PE but not 7-AAD were early apoptotic, whereas those were Annexin V-PE and 7-AAD positive were late apoptotic or necrotic.

### Statistical analysis

SPSS 22 (Chicago, Illinois, U.S.A.) was used for statistical analyses and data were presented as mean ± S.D. Correlations between expressions of *CRP* and *ATG9B* and the clinical-pathological characteristics were analyzed using two-sided Fisher’s exact test. The correlation between the protein expressions of *CRP* and *ATG9B* was assessed using Spearman’s rank correlation coefficient test. The Kaplan–Meier method was applied to draw OS curves and the expression comparisons distinction between groups was evaluated using the log-rank test. *P*<0.05 was considered statistically significant.

## Results

### The expression of *CRP* and *ATG9B* in serum and tissues

The concentration of CRP in human serum was evaluated using ELISA method. The results showed that the expression of CRP in CCRCC group was significantly higher than that in control group (<10 mg/l, Figure 1A). Meanwhile, amongst 185 CCRCC serum samples, there were high expressions of serum CRP in 159 cases (>30 mg/l), moderate expression of CRP in 18 cases (11–30 mg/l), and low expression of CRP in 8 cases (<10 mg/l).

**Figure 1:** *CRP* and *ATG9B* expression in tissues and the relationship between *CRP* expression and OS rate of patients (**A**) Serum *CRP* protein was lowly expressed in patients of the normal group, but highly expressed (>30 mg/l) in 159 CCRCC cases, medium expressed in 18 CCRCC cases (11–30 mg/l) and lowly expressed (<10 mg/l) in 8 CCRCC cases. (**B**) *ATG9B* expression in all normal kidney and tumor tissues was positive, with 82 lowly expressed and 103 highly expressed in CCRCC patients group. The positive signal is in the cancer cell cytoplasm. (**C**) Patients with high *CRP* expression level had worse survival outcomes compared with low expression group. *P<0.05 compared with control group.

The IHC staining results showed that compared with adjacent tissues, CCRCC tissues demonstrated more positive expression of ATG9B. In CCRCC tissues, low expression of ATG9B was detected in 82 patients and highly expressed ATG9B was observed in 103 patients (Figure 1B). The positive signal was in the cytoplasm of cancer cells.

### The correlation between gene expression and the pathological characteristics of CCRCC patients

The relationship between *CRP* and *ATG9B* expression levels and CCRCC patients’ characteristics were analyzed using two-sided Fisher’s exact test. As was shown in Table 2, high expression of *CRP* or *ATG9B* was positively related to advanced TNM stage and distant metastases. In addition, there was also a positive correlation between *CRP* expression and *ATG9B* expression (Table 3).

**Table 2:** Associations between expressions of CRP and ATG9B and clinicopathologic characteristics in CCRCC patients

Characteristics	Volume (%)	CRP expression (*n*=185)		*P*	ATG9B expression (*n*=185)		*P*
		Low (*n*=97) (%)	High (*n*=88) (%)		Low (*n*=82) (%)	High (*n*=88) (%)	
Age (years)							
≤52	73 (39.46)	36 (49)	37 (51)	0.548	38 (52)	35 (48)	0.097
>52	112 (60.54)	61 (55)	51 (45)		44 (39)	68 (61)	
Gender							
Male	105 (56.76)	52 (49)	53 (51)	0.377	51 (49)	54 (51)	0.232
Female	80 (43.24)	45 (56)	35 (44)		31 (39)	49 (61)	
Histologic grade							
Grade 1–2	77 (41.62)	39 (51)	38 (49)	0.765	37 (48)	40 (52)	0.453
Grade 3–4	108 (58.38)	58 (54)	50 (46)		45 (42)	63 (58)	
TNM stage							
I–II	98 (52.97)	60 (61)	38 (39)	**0.013**	32 (33)	66 (67)	**0.001**
III–IV	87 (47.03)	37 (43)	50 (57)		50 (57)	37 (43)	
Distant metastasis							
Absent	127 (68.65)	75 (59)	52 (41)	**0.011**	63 (49)	64 (51)	**0.038**
Present	58 (31.35)	22 (38)	36 (62)		19 (33)	39 (67)	

*P*; Bold values mean significant results

**Table 3:** Correlations between CRP and ATG9B

Spearman’s rho		CRP	ATG9B
CRP	Correlation coefficient	1.000	0.850
	Sig. (two-tailed)	0.000	0.000
ATG9B	Correlation coefficient	0.850	1.000
	Sig. (two-tailed)	0.000	0.000

### The correlation between *CRP* expression and patients’ prognosis

Survival curves were generated by means of the Kaplan–Meier method and the distinctions amongst groups with different expressions were detected using the log-rank test. The correlation between *CRP* expression level and OS of CCRCC patients was shown in Figure 1C. The results indicated that patients with high *CRP* expression level had a lower OS and poorer prognostic result than those who with low *CRP* expression level.

### The correlation between *CRP* expression and *ATG9B* expression

The effect of siRNA transfection on the expression of *CRP* was confirmed by RT-qPCR (Figure 2A). Compared with the negative control group, siRNAs (siRNA-1 and siRNA-2) could significantly inhibit *CRP* mRNA expression. *ATG9B* expression dramatically decreased after the transfection of siRNAs. In addition, the expression level of *ATG9B* decreased more quickly than that of *CRP* (Figure 2B). According to Western blot results, the expression levels of *CRP* and *ATG9B* proteins were remarkably down-regulated.

**Figure 2:** *CRP* silences effects and its correlation with *ATG9B* expression (**A**) siRNAs could significantly down-regulate mRNA expressions of *CRP* and *ATG9B* protein. mRNA levels of *CRP* and *ATG9B* were both significantly lower in siRNA-1 and siRNA-2 groups than in control group. (**B**) *CRP* protein level as well as *ATG9B* protein level in siRNA-1 and siRNA-2 groups was much lower than in control group. *P<0.05, ^#^*P*<0.05 compared with control group.

### The inhibitive effects of *CRP* on the apoptosis of 786-O cells

The results of Hoechst 33258 staining of the tumor cell cytoplasm showed that the transfection of siRNAs significantly promoted the apoptosis in 786-O cells (Figure 3A). Annexin-V and 7-AAD dual-staining FCM results demonstrated that the apoptosis rate of cells in siRNA-1 or siRNA-2 group was much higher than that in the control group (Figure 3B). This also indicated that the apoptosis of 786-O cells could be induced through silencing *CRP* expression. On the other hand, cell cycle assay also demonstrated that cells were arrested in G_1_-phase in the two siRNA groups (Figure 3C).

**Figure 3:** Inhibition of *CRP* expression induces cell cycle arrest and the apoptosis in 786-O cells (**A**) The apoptosis of 786-O cells increased by either siRNA by ~2.5 times. Scale bar: 30 μm. (**B**) Dual-staining FCM test results showed that apoptotic cells transfected with siRNAs were much more than those in the control group. * means *P*<0.05 compared with the control group. (**C**) The cell cycle was significantly arrested in G_0_/G_1_-phase in siRNA groups. *P<0.05 compared with control group.

### The synchronous expression of *CRP* expression and *ATG9B* expression

As shown in Figure 4, mRNA expression levels of *CRP* and *ATG9B* in overexpressed group was up-regulated by more than twice in comparison with the control group. Western blot results revealed that overexpression of *CRP* could significantly up-regulate the expression of *ATG9B*.

**Figure 4:** The effects of *CRP* overexpression and its correlation with *ATG9B* expression (**A**) *CRP* mRNA expression increased by ~2.5 times, while *ATG9B* expression increased by ~2.2 times significantly in *CRP* overexpression group than in Scr group. (**B**) CRP level increased significantly because of its overexpression, which also improved ATG9B level. *P<0.05, ^#^*P*<0.05 compared with Scr group.

### The inhibitive effects of *CRP* expression on the apoptosis in 786-O cells

The apoptotic rate of the overexpression group presented a drastic decline in comparison with negative control group, which also suggested that *CRP* overexpression could inhibit apoptosis (Figure 5A). Moreover, *CRP* expression group displayed much fewer apoptotic cells than the negative control group, shown by Annexin-V and 7-AAD dual-staining FCM test results. *CRP* overexpression could suppress cell apoptosis (Figure 5B). S- and G_2_/M-phases increased in 786-O cells of overexpression group compared with the negative control group (Figure 5C). This showed that *CRP* expression level could exert influence on the cell cycle of 786-O cells.

**Figure 5:** *CRP* overexpression promotes the apoptosis of 786-O cells and reduces the cell cycle (**A**) 786-O cell apoptosis decreased by approximately two-fold. Scale bar: 30 μm. (**B**) the number of apoptotic cells was much less in CRP overexpression group than that in Scr group. (**C)** The percentage of cells that were arrested in G_0_/G_1_-phase in CRP overexpression group was reduced significantly compared with Scr group. *P<0.05 compared with Scr group.

## Discussion

In the present study, we have discovered that the expression of *CRP* and *ATG9B* is significantly correlated with CCRCC TNM staging, metastasis, and OS. A higher level of *CRP* indicates a poorer OS of CCRCC patient. The inhibition of *CRP* expression significantly increased the apoptosis and cell cycle arrest of CCRCC cell line 786-O. *CRP* expression is positively correlated with *ATG9B*, and its overexpression leads to less apoptosis and less cell cycle arrest of 786-O cells. CCRCC is the most common kind of RCC with poor prognosis with a 5-year survival rate of 0–10% [27]. To understand the relationship of *CRP* and *ATG9B* expression and CCRCC are significant to the development of CCRCC prognosis and treatment.

In our study, we found that *CRP* expression was associated with *ATG9B* expression. The inhibition of *CRP* expression was accompanied by a decreased expression of *ATG9B* and the overexpression of *CRP* was accompanied with an increased expression of *ATG9B*. Serum *CRP* protein was lowly expressed in normal patients. Amongst CCRCC patients, 159 were found with high-level *CRP* (>30 mg/l), 18 medium-level (11-30 mg/l), and 8 low-level (<10 mg/l). On the other hand, *ATG9B* was found overexpressed in most of CCRCC patients. *CRP* was found significantly associated with OS of CCRCC patients. Based on the above results, we speculated that the expression of *CRP* and *ATG9B* was positively correlated with CCRCC and it may indicate a poorer status of CCRCC. Our results are consistent with previous studies, in which identical findings were demonstrated in regards of RCC OS and aberrant *CRP* expression [17,28–30]. Thus, we speculated that the aberrant overexpression of *CRP* and *ATG9B* could possibly promote CCRCC development.

The *in vivo* experiment results support our hypothesis that the aberrant overexpression of *CRP* and *ATG9B* could promote CCRCC development, possibly by influencing the cell cycle and apoptosis. The inhibition of *CRP* expression promoted whereas the promotion of *CRP* expression inhibited 786-O cell cycle arrest and apoptosis. As a stable downstream inflammation marker, it can be stimulated by IL-1 and tumor necrosis factors (TNFs) [31]. Chronic inflammation can be predictor of cancer initiation, progression, metastasis, and survival. *CRP*-level measurements can be clinically significant for RCC prognosis [32,33]. Hence, we inferred that *CRP* could be involved in CCRCC development via some inflammation pathway that involves ILs and TNFs and affect CCRCC cell proliferation and apoptosis.

On the other hand, *CRP* overexpression was found to be accompanied/associated with *ATG9B* overexpression. *ATG9B* is involved in autophagy process that delivers cytoplasmic constituents degraded by autophagosomes to lysosomes for digestion [34], which is a common scene during carcinogenesis [26]. Autophagy can play a protective role in tumor cell survival, and can also contribute to cancer progression by preventing tumor cell from programming death [35]. Zhang et al. [21] found aberrant promoter methylation of *ATG9B* in sporadic breast carcinoma. Oncogenic autophagy in CCRCC was reported to be regulated by some molecules, which could contribute to the CCRCC progression [25]. *ATG* genes as well as ATG-interacting genes have been reported to be related to the development of diverse carcinomas such as lung cancer and CCRCC etc. [36]*.* Based on the previous findings as well as ours, we speculated that aberrant *ATG9B* expression might contribute to the aberrant autophagy of CCRCC cells, which then induced CCRCC progression.

Certain limitations exist in the present study. First of all, *in vivo* studies need to be done to elaborate the role of *CRP* and *ATG9B* expression during CCRCC development. Second, *ATG9B*-related autophagy pathway can be further studied for a better comprehension of the *ATG9B*-related mechanism of CCRCC pathogenesis. Third, the influence between *CRP*-related inflammation pathways and CCRCC need to be further explored. Fourth, *in vivo* experiments need to be further studied to verify the *in vitro* discoveries. Last, detailed correlation between *ATG9B* and CCRCC pathogenesis need further investigation as well.

In conclusion, our study showed that *CRP* and *ATG9B* were both aberrantly overexpressed in CCRCC tissues and cells, and they were closely correlated with CCRCC TNM staging, metastasis, and OS. The suppression of *CRP* expression led to the cancer cell cycle arrest and apoptosis. The results indicate that *CRP* and *ATG9B* could be significant predictors of CCRCC and can be a valuable target for CCRCC therapy.

## Supporting information

**Table S1:** SiRNA sequences that were used in the experiments.

## Abbreviations

ATG9B: autophagy-related 9B
CCRCC: clear cell renal cell carcinoma
CRP: C-reactive protein
DMEM: Dulbecco’s modified Eagle’s medium
FCM: flow cytometry
IHC: immunohistochemistry
OS: overall survival
RCC: renal cell carcinoma
RT-qPCR: real-time quantitative PCR
TNF: tumor necrosis factor
